# Efficacy of Gamma Globulins in Children with Kawasaki Disease and Factors Influencing Children's Short-Term Prognosis

**DOI:** 10.1155/2022/5137874

**Published:** 2022-07-30

**Authors:** Hao Sun, Huimin Lu, Yunhong Wu

**Affiliations:** Department of General Paediatrics, Children's Hospital of Shanxi, Taiyuan City, 030000 Shanxi, China

## Abstract

**Purpose:**

To explore and analyze the therapeutic effect of gamma globulins (GG) on Kawasaki disease (KD) in children and the influencing factors of short-term prognosis.

**Methods:**

First, 90 pediatric KD patients admitted between January 2019 and January 2021 were selected and divided into a control group (*n* = 40) and a research group (*n* = 50) according to the difference in treatment. In addition to routine treatment and nursing given to both groups, control group was given aspirin (ASA), based on which research group was supplemented with GG therapy. The treatment outcome and adverse events (AEs) of the two cohorts of patients were analyzed and compared, and the influencing factors of children's short-term prognosis were analyzed by logistics multivariate analysis.

**Results:**

Research group had a statistical higher overall response rate than control group, with significantly fewer cases suffering from AEs such as nausea and vomiting, diarrhea, rash, dizziness and headache, and coronary artery injury. On the other hand, logistics multivariate analysis identified that gender, body mass index (BMI), onset time, platelet (PLT), and treatment mode all independently influence the short-term prognosis of children with KD.

**Conclusions:**

GG therapy is effective in treating pediatric KD patients and can effectively prevent AEs. In addition, gender, BMI, onset-to-treatment time, PLT, C-reactive protein (CRP), and treatment methods are independent risk factors for short-term prognosis of children with KD.

## 1. Introduction

Kawasaki disease (KD) is an acute systemic vasculitis with complex pathological triggers, usually occurring in children under the age 5 [1]. According to KD epidemiological data, the median diagnosis age of the disease is 1.4 years old, with a predilection for boys and the rainy season as the peak period [2]. The disease mainly has a negative impact on children's medium-sized arteries, especially the coronary arteries [3]. The main clinical presentations of KD are fever, rash, cervical lymph node enlargement, and oral mucosal erythema [4]. For pediatric KD patients, delayed treatment and intervention can result in 25% of them developing coronary artery injury that may consequently lead to adverse events (AEs) such as coronary artery aneurysm, ischemic heart disease, or sudden death [5, 6]. Therefore, optimizing treatment strategies for pediatric KD patients is of great significance for improving patient prognosis and optimizing clinical management of the disease.

Though not completely clarified, the pathological mechanism of KD is shown to be associated with immune system activation and inflammatory cascade caused by unknown stimuli [7]. Aspirin (ASA), or acetylsalicylic acid, in combination with gamma globulins (GG), constitutes a key part of the standard treatment plan for KD, which can exert synergistic systemic anti-inflammatory effects and reduce coronary artery injury [8, 9]. ASA is known to induce the production of some proresolving lipid-derived mediators, the secretion of which is used by the immune system to control the inflammatory response associated with injury stimuli, endowing ASA with anti-inflammatory effects [10]. Additionally, it has analgesic, antipyretic, and antiplatelet pharmacological actions [11]. GG, on the other hand, is an immunoglobulin G (IgG) mixed preparation made from the plasma purification of thousands of healthy donors, which can be used to treat autoimmune diseases and inflammatory diseases [12]. GG is shown to exert anti-inflammatory effects via blocking Fc receptors, neutralizing pathogenic products of unknown infectious agents, and regulating inflammatory cytokines [13].

Considering that the curative effect of GG therapy in children with KD and the influencing factors of children's short-term prognosis have not been fully clarified, this research conducts relevant analyses to provide new insights into the treatment of pediatric KD.

## 2. Data and Methods

### 2.1. General Data

This research, ratified by Children's Hospital of Shanxi Ethics Committee, enrolled 90 children with KD from January 2019 to January 2021 and assigned them to a control group (*n* = 40) and a research group (*n* = 50) according to the difference in treatment. In addition to routine treatment and nursing in both groups, control group was given ASA, based on which research group was supplemented with GG therapy. Control group comprised 25 boys and 15 girls, aged 2.47 ± 0.90 years, with the onset-to-treatment time of 6.57 ± 1.55 days. Research group had 30 boys and 20 girls, aged 2.43 ± 1.47 years, with the onset-to-treatment time of 6.90 ± 1.52 days. The two cohorts showed no distinct differences in baseline data (*P* > 0.05). All subjects' legal guardians were fully informed of the purpose of the study and provided informed consent.

### 2.2. Inclusion and Exclusion Criteria

All the included children had confirmed the first episode of KD and met the indications of GG and ASA, with normal growth and development and intact medical records.

Children were excluded from this study if they had infectious diseases, rash and fever illness, vital organ-associated diseases, congenital heart disease, chronic obstructive pulmonary disease, or drug allergies.

### 2.3. Treatment Methods

Children in control group were given 30-50 mg/kg ASA (Beijing Kangruina Biotechnology Co., Ltd., A1189) that was divided into 2-3 oral doses every day. The dose was gradually reduced after the body temperature recovered for 3 days. About 2 weeks after treatment, ASA was reduced to 3-5 mg/kg per day and administered orally for 6-8 weeks.

Research group was given intravenous GG (Shanxi Kangbao Biological Products Co., Ltd., S19994004) in addition to the above treatment, that is, 1.0 g/kg/d GG was given 5 days after the onset of the disease with the infusion time of 8-12 h, for 2 days.

### 2.4. Curative Effect Evaluation

If the child's symptoms such as fever, lymph node swelling, congestion of conjunctiva, and pharyngeal mucosa disappear, and the area of macula recovers by 90% or more, it is regarded as cured; if the above-mentioned symptoms disappear and the macula area recovers by 75-89%, it is considered markedly effective; if the child's symptoms have improved but not completely disappeared, with the macula area recovered by 30-74%, it is considered effective; if the child has no change in the above symptoms with the macula area recovered <30%, it was regarded as ineffective.

### 2.5. Outcome Measures

#### 2.5.1. Curative Effect

The corresponding cases of cured, effective, effective, and ineffective patients were recorded according to the above evaluation criteria, and the percentage of the sum of cured, effective, and effective in the total cases was the total effective rate.

#### 2.5.2. Incidence of AEs

The incidence of AEs (chills, nausea and vomiting, dizziness, and headache) was recorded.

#### 2.5.3. Coronary Artery Injury

Coronary artery injury of children was evaluated by echocardiography, and the incidence of mild, moderate, and severe coronary artery injury and the total incidence were recorded. The criteria are as follows: mild injury: coronary artery diameter 2.5-4.0 mm; moderate injury: coronary artery diameter 4.0-6.0 mm; severe injury: coronary artery diameter ≥7mm.

#### 2.5.4. Short-Term Prognosis

Events such as ineffective treatment, adverse reactions, and coronary artery injury during treatment were considered as poor short-term outcomes.

The primary outcome measures of this study are curative effect and incidence of adverse reactions, and the secondary ones are coronary artery injury and short-term outcome.

### 2.6. Statistical Analysis

We analyzed the data and obtained corresponding pictures with GraphPad Prism 6 (GraphPad Software Inc., USA). The enumeration data, recorded as the number of cases/percentage (n/%), were analyzed via the chi-square test or the chi-square continuity correction when the theoretical frequency of the former test was below 5. Mean ± SEM was used to indicate the measurement data, and the independent sample *t*-test was used for comparison of data between groups. Univariate and multivariate analyses of independent risk factors affecting the short-term prognosis of children with KD were performed using the SPSS Regression SPSS22.0 (SPSS, Inc., Chicago, IL, USA) models. *P* < 0.05 was the statistical significance level for all tests in this study.

## 3. Results

### 3.1. Baseline Data of Pediatric KD Patients

By analyzing the general data of 90 pediatric KD patients (Table 1), we found that control group and research group had no statistical difference in sex, age, onset-to-treatment time, duration of fever, body temperature, KD type, overweight, platelet (PLT), C-reactive protein (CRP), alanine aminotransferase (ALT), and aspartate aminotransferase (AST), which were comparable (*P* > 0.05).

### 3.2. Therapeutic Effect of Pediatric KD Patients

We analyzed the curative effect of two groups to evaluate the influence of the two interventions on KD patients. According to the data (Table 2), the cure rate of research group was 34.00% that of the control group (22.50%). In addition, the total effective rate was 90.00% in the research group and 72.50% in the control group, with statistical significance between them (*P* < 0.05).

### 3.3. Incidence of AEs in Pediatric KD Patients

We compared and analyzed the incidence of AEs in terms of chills, nausea and vomiting, dizziness, and headache and found that the total incidence was significantly lower in research group compared with control group (4.00% vs. 25.00%, *P* < 0.05; Table 3).

### 3.4. Incidence of Coronary Artery Injury in Pediatric KD Patients

We also recorded the occurrence of coronary artery injury in both groups of KD patients, so as to compare and analyze the influence of the two interventions on coronary artery injury. The results revealed that more patients in control group suffered from coronary artery injury of various severity, with a higher overall incidence compared with research group (22.50% *vs.* 4.00%, *P* < 0.05). See Table 4.

### 3.5. Analysis of Influencing Factors of Short-Term Prognosis of Pediatric KD Patients

The influencing factors of short-term prognosis in 90 pediatric KD patients were analyzed by univariate analysis. The data showed that the adverse factors significantly affecting the short-term prognosis of children with KD included sex, onset-to-treatment time, overweight, PLT, CRP, and treatment methods (*P* < 0.05). Multivariate logistic regression analysis further confirmed that gender, onset-to-treatment time, overweight, PLT, CRP, and treatment mode were significantly and independently associated with poor short-term prognosis of children with KD (*P* < 0.05; Tables 5 and 6).

## 4. Discussion

KD, as a self-limiting childhood disease, can be divided into complete KD and incomplete KD, in which the former meets the diagnostic criteria of KD, while the latter does not fully meet [14]. This may lead to difficult diagnosis and delayed treatment in children with incomplete KD, increasing the risk and mortality of coronary artery aneurysm, myocardial suppression, arrhythmia, and other diseases [15]. The etiology of KD remains to be defined and may be related to respiratory disease-associated pathogens such as coronavirus, rhinovirus, and adenovirus [16]. This report mainly analyzes the curative effect and short-term prognosis of children with KD, hoping to make a contribution to optimizing the treatment and improving the prognosis of KD.

This research included 90 pediatric KD patients who were assigned to the control group treated with ASA and the research group additionally treated with GG. In our study, the total effective rate of treatment was obviously higher in research group than in control group (90.00% vs. 72.50%), indicating that GG intervention can significantly improve the clinical efficacy of children with KD. In addition, 10.00% of the children in research group did not respond to GG therapy and had GG resistance, which was consistent with the report of McCrindle et al. [17]. In terms of safety, chills, dizziness, and headache were the main AEs in control group versus chills alone in research group; the overall incidence of AEs was obviously lower in research group compared with control group (4.00% vs. 25.00%), suggesting that in treating pediatric KD patients, GG has a certain safety that is better than ASA alone. Mohammadzadeh et al. [18] reported that GG combined with ASA reduced the complication rate from 47% at the onset of pediatric KD to 7% at the sixth month, similar to our findings. In the evaluation of coronary artery injury, research group was found with fewer cases of mild, moderate, and severe coronary artery injury and a notably lower overall incidence compared with control group (4.00% vs. 22.50%). In the research of Galeotti et al. [12], GG effectively prevented KD complicated artery injury in children and reduced the risk of coronary artery disease from as high as 25% to 2-4%, which is consistent with our research results. Coronary artery injury is mainly attributed to KD, accompanied by thrombosis and distal embolism, for which ASA, an antithrombotic drug, shows some certain preventive effect [19]. Finally, we confirmed through univariate and multivariate logistic regression analyses that gender, onset-to-treatment time, overweight, PLT, and treatment methods were independent risk factors for poor short-term prognosis of children with KD, similar to the results of Qiu et al. [20]. The report of Huang et al. [21] confirmed that PLT, CRP, neutrophil percentage, serum albumin, serum sodium, etc. were the risk factors of GG resistance in children with KD, which confirms the accuracy of our findings. Hu and Ren [22] also pointed out that immunoglobulin M (IgM), IgA, and the number of coronary arteries involved (NCAI) are the adverse prognostic factors of coronary artery injury in children with KD.

The novelty of this study lies in that it demonstrates the effectiveness and safety of GG treatment in children with KD from the perspectives of efficacy and incidence of adverse reactions and confirms that GG treatment has a certain protective effect on the prognosis of children with KD from the aspects of the occurrence of coronary artery injury and the short-term prognostic factors. The above provides new insights into the management optimization of pediatric patients with KD. However, there are still some limitations. First, it is a single-center research, which is prone to information bias. Second, the basic experimental analysis of related therapeutic mechanisms can be supplemented to further clarify the anti-KD mechanism of GG and the prevention mechanism of KD-related coronary artery injury. Finally, if children's long-term prognosis can be discussed in future research, the influence of the two intervention methods on the long-term prognosis of children with KD will be further understood. We will continue to improve the research project from the above aspects.

## 5. Conclusion

Our data indicate that GG treatment is effective in the treatment of children with KD, which can effectively reduce the incidence of AEs and help prevent coronary artery injury. On the other hand, the poor short-term prognosis of some children with KD may be related to factors such as sex, onset-to-treatment time, overweight, PLT, and treatment methods. In clinical practice, reasonable intervention measures can be formulated according to the above factors to improve the short-term prognosis of children with KD.

## Figures and Tables

**Table 1:** Baseline data of pediatric KD patients [*n*, mean ± SEM].

Factor	Control group (*n* = 40)	Research group (*n* = 50)	*χ* ^2^/*t*	*P*
Gender (male/female)	25/15	30/20	0.058	0.809
Age (years old)	2.47 ± 0.90	2.43 ± 1.47	0.151	0.880
Onset-to-treatment time (d)	6.57 ± 1.55	6.90 ± 1.52	1.015	0.313
Duration of fever (d)	3.37 ± 0.72	3.60 ± 0.74	1.483	0.142
Body temperature (°C)	38.90 ± 0.45	39.09 ± 0.71	1.472	0.145
Type of KD (complete/incomplete)	18/22	25/25	0.223	0.637
Overweight (yes/no)	27/13	40/10	1.825	0.177
PLT (10^9/L)	372.49 ± 124.89	379.80 ± 141.42	0.257	0.798
CRP (mg/L)	76.07 ± 16.35	82.41 ± 18.02	1.728	0.088
ALT (U/L)	35.45 ± 11.76	35.94 ± 13.68	0.180	0.858
AST (U/L)	32.89 ± 17.45	34.90 ± 14.51	0.597	0.552

**Table 2:** Therapeutic effect of pediatric KD patients [*n* (%)].

Groups	*n*	Cured	Markedly effective	Effective	Ineffective	Total effective rate (%)
Control group	40	9 (22.50)	12 (30.00)	8 (20.00)	11 (27.50)	29 (72.50)
Research group	50	17 (34.00)	15 (30.00)	13 (26.00)	5 (10.00)	45 (90.00)
*χ* ^2^ value	—	—	—	—	—	4.656
*P* value	—	—	—	—	—	0.031

**Table 3:** Incidence of adverse events in pediatric KD patients [*n* (%)].

Categories	Control group (*n* = 40)	Research group (*n* = 50)	*χ* ^2^ value	*P* value
Chills	5 (12.50)	2 (4.00)	—	—
Nausea and vomiting	1 (2.50)	0 (0.00)	—	—
Dizziness and headache	4 (10.00)	0 (0.00)	—	—
Total incidence	10 (25.00)	2 (4.00)	8.481	0.004

**Table 4:** Incidence of coronary artery injury in pediatric KD patients [*n* (%)].

Categories	Control group (*n* = 40)	Research group (*n* = 50)	*χ* ^2^ value	*P* value
Mild	4 (10.00)	2 (4.00)	—	—
Moderate	3 (7.50)	0 (0.00)	—	—
Severe	2 (5.00)	0 (0.00)	—	—
Total incidence	9 (22.50)	2 (4.00)	7.089	0.008

**Table 5:** Assignment of logistic multivariate regression analysis.

Factors	Variables	Assignment
Sex	X1	Male = 0, female = 1
Age (years old)	X2	Continuous variable
Onset-to-treatment time (d)	X3	Continuous variable
Fever time (d)	X4	Continuous variable
Body temperature (°C)	X5	Continuous variable
KD type	X6	Complete = 0, incomplete = 1
Be overweight	X7	Yes = 0, no = 1
PLT (10^9/L)	X8	Continuous variable
CRP (mg/L)	X9	Continuous variable
ALT (U/L)	X10	Continuous variable
AST (U/L)	X11	Continuous variable
Treatment methods	X12	Aspirin = 0, aspirin + GG = 1

**Table 6:** Univariate and multivariate logistic analysis of short-term prognosis of pediatric KD patients.

Characteristic	Univariate		Multivariate	
	OR (95% CI)	*P*	OR (95% CI)	*P*
Sex	1.304 (1.039-1.632)	0.024	2.113 (1.354-3.304)	0.002
Age (years old)	2.034 (0.960-1.547)	0.068		
Onset-to-treatment time (d)	2.315 (1.124-4.875)	0.023	2.279 (1.290-4.061)	0.007
Duration of fever (d)	2.109 (0.926-4.453)	0.057		
Body temperature (°C)	1.556 (0.913-2.684)	0.114		
Types of KD	1.009 (0.987-1.003)	0.356		
Overweight	2.872 (1.425-4.826)	<0.001	1.854 (1.013-3.397)	0.045
PLT (10^9/L)	2.541 (1.149-3.751)	<0.001	2.105 (1.127-3.915)	0.019
CRP (mg/L)	2.213 (1.123-3.985)	0.009	2.319 (1.305-4.228)	0.005
ALT (U/L)	1.011 (0.008-1.750)	0.525		
AST (U/L)	1.058 (0.356-1.167)	0.308		
Treatment methods	3.754 (1.319-10.522)	0.012	3.061 (2.245-5.467)	0.029

## Data Availability

The labeled dataset used to support the findings of this study are available from the corresponding author upon request.
